# *Rice stripe virus* p2 Colocalizes and Interacts with *Arabidopsis* Cajal Bodies and Its Domains in Plant Cells

This article has been retracted.

**DOI:** 10.1155/2020/5182164

**Published:** 2020-06-16

**Authors:** Luping Zheng, Pengxiang Hong, Xiaonan Guo, Yang Li, Li Xie

**Affiliations:** ^1^Key Laboratory of Biopesticide and Chemical Biology, Ministry of Education, Fujian Agriculture and Forestry University, Fuzhou 350002, China; ^2^College of Plant Protection, Fujian Agriculture and Forestry University, Fuzhou 350002, China

## Abstract

p2 of *rice stripe virus* may translocate from the nucleus to the cytoplasm and recruit nucleolar functions to promote virus systemic movement. Cajal bodies (CBs) are nuclear components associated with the nucleolus, which play a major role in plant virus infection. Coilin, a marker protein of CBs, is essential for CB formation and function. Coilin contains three domains, the N-terminal, the center, and the C-terminal fragments. Using yeast two-hybrid, colocalization, and bimolecular fluorescence complementation (BiFC) approaches, we show that p2 interacts with the full-length of *Arabidopsis thaliana* coilin (Atcoilin), the center and C-terminal domain of Atcoilin in the nucleus. Moreover, the N-terminal is indispensable for Atcoilin to interact with Cajal bodies.

## 1. Introduction

Plant viruses invade plants by infecting host cell to complete replication. The replicated viruses then infect more cells to cause virus diseases. The nucleus is a significant cell organelle for virus infection. An increasing number of plant viruses are reported to interact with the nucleus and its compartments. Cajal bodies (CBs) are distinct nuclear bodies physically and functionally associated with the nucleolus [1]. Virus may rearrange CBs to obtain energy for virus replication or virus pathogenicity [2, 3]. Coilin is a critical protein of CBs; many viruses were reported to bind with coilin to finish viral infection. Coilin serves to increase virus pathogenicity; *Groundnut rosette virus* (GRV) ORF3 protein hijacks CBs as vehicles to enter the nucleolus in virus systemic infection [4, 5]; *herpes simplex virus* 1 and *adenoviruses* relocalize coilin and other CB components around viral replication centers [2]. TGBp1 encoded by *Poa semilatent virus* (PSLV) relocalized with coilin in the cytoplasm resulting in the inclusions of various sizes [6]. However, coilin also contributes to plant defense against virus, such as *tobacco rattle virus* and *tomato black ring virus* [1]. Coilin usually comprises three protein domains: the N- and C-termini are highly conserved, while the middle portion is not conserved.

*Rice stripe virus* (RSV) is an important rice virus in Asia, causing great rice yield losses [7, 8]. RSV is the type species of genus *Tenuivirus*, but has not been assigned to any family [9]. It is transmitted by the small brown plant hopper (*Laodelphax striatellus* Fallén) in a persistent and circulative-propagative manner [10]. The genome of RSV contains four single-stranded RNAs (ssRNAs), which were named RNA1-RNA4 in the decreasing order of size [11]. RNA1 is a negative sense and encodes RNA-dependent RNA polymerase (RdRp) [12]. RNA2-RNA4 employ an ambisense coding strategy, each encode two proteins, one in the virus-sense strand (vRNA) named p2-p4, respectively, and the other in the virus complementary-sense strand (vcRNA) named pc2-pc4 respectively [10]. p4 is a nonstructural disease-specific protein, which often reaches a high level in RSV-infected plants [13]; pc4 is a movement protein playing roles in virus pathogenicity [14, 15]. p3 is a silencing suppressor [16], and pc3 is a nucleocapsid protein [17]. pc2 shares many characteristics to the glycoproteins [18]. p2 is another silencing suppressor and interacts with fibrillarin to promote virus systemic movement [19, 20]. Fibrillarin is a major nucleolus protein, localized in nucleolus and CBs; CBs are often physically and functionally associated with the nucleolus to play a significant role in modulating some virus infections [1, 2], for example, GRV finished its systemic infection via a mechanism involving the reorganization of CBs and their fusion with the nucleolus [4]. p2 is a nuclear-cytoplasmic trafficking protein, it may recruit Cajal bodies to involve in RSV infection.

In this study, the interactions between p2 and the full length of coilin from *Arabidopsis thaliana* (Atcoilin) and between p2 and the three functional domains of Atcoilin are identified through yeast two-hybrid (Y2H), colocalization, and BiFC methods. The results indicated that p2 interacts with the full-length Atcoilin, the center and C-terminal domains of Atcoilin in the nucleus, but not interacts with the N-terminal domain.

## 2. Results

### 2.1. p2 Interacts with *Atcoilin* in Y2H Assay

Atcoilin contains three functional domains, an N-terminal ordered domain (NOD, Atcoilin-1), a central disordered domain (IDD, Atcoilin-2), and a C-terminal domain (CTD, Atcoilin-3) (Figure 1). To perform Y2H assay, the full-length ORF of p2 was cloned into the vector pGADT7 (pGAD), creating pGAD-p2; the full-length ORF of Atcoilin and the three domains of Atcoilin (Atcoilin-1, Atcoilin-2, and Atcoilin-3) were inserted into the vector pGBKT7 (pGBK), creating pGBD-Atcoilin, pGBD-Atcoilin1, pGBD-Atcoilin2, and pGBD-Atcoilin3. The same amount of yeast cells was resuspended in 20 *μ*L of sterile water and diluted in sterile water at ratios of 1 : 1, 1 : 10, and 1 : 100. As shown in Figure 2, yeast cells cotransformed with pGAD-p2/pGBK-Atcoilin, pGAD-p2/pGBK-Atcoilin2, and pGAD-p2/pGBK-Atcoilin3 grew on SD medium lacking adenine (Ade), histidine (His), leucine (Leu), and tryptophan (Trp) (SD/Trp-Leu-His-Ade-), while cotransforms of pGAD-p2/pGBK-Atcoilin1, pGBK-p2/pGAD, pGBK/pGAD-Atcoilin, pGBK/pGAD-Atcoilin1, pGBK/pGAD-Atcoilin2, and pGBK/pGAD-Atcoilin3 failed to grew on SD/Trp-Leu-His-Ade-. Cotransforms of pGAD-T/pGBK-53 and pGAD-T/pGBK-Lam were individually used as positive controls and negative controls. These results indicated that p2 of RSV interacts with full-length of Atcoilin, in which the central disordered domain and the C-terminal domain are involved in their interaction.

### 2.2. p2 Colocalizes with Atcoilin

In colocalization assay, the full-length ORF of p2 was cloned into pEarleyGate102 (CFP) and that of Atcoilin, Atcoilin1, Atcoilin2, and Atcoilin3 into pEarleyGate101 (YFP). *Agrobacterium tumefaciens* (*A. tumefaciens*) EHA105 carrying each of these constructs were mixed and infiltrated into the leaves of *Nicotiana benthamiana* (*N. benthamiana*). As shown in Figure 3, p2 and Atcoilin colocalize in the nucleolus and Cajal bodies, p2 and Atcoilin2 and p2 and Atcoilin3 can also colocalize to the nucleus, but p2 fails to colocalize with Atcoilin1.

### 2.3. p2 Binds to Atcoilin in BiFC Assay

In BiFC assay, the full-length ORF of p2 was cloned into pEarley201-YC (YC) and that of Atcoilin, Atcoilin1, Atcoilin2, and Atcoilin3 into pEarley201-YN (YN). *A. tumefaciens* EHA105 carrying each of these constructs were mixed and infiltrated into leaves of *N. benthamiana*. As shown in Figure 4, strong yellow fluorescent was detected in the nucleus of *N. benthamiana* leaf epidermal cells when YC-p2 individually mixed with YN-Atcoilin, YN-Atcoilin2, or YN-Atcoilin3. However, none can be found in the *N. benthamiana* leaf epidermal cells coinfiltrated by YC-p2 and YN-Atcoilin1. This confirms the results in Y2H assays, p2 interacts with the full-length of Atcoilin, the central domain Atcoilin2, and the C-terminal domain Atcoilin3, except the N-terminal domain Atcoilin1.YN and YC were also mixed and infiltrated, no fluorescent was detected (data not shown).

## 3. Discussion

Coilin has low homology in amino acid sequences in different species, but coilin of different organisms demonstrate a high level of structural similarity, such that their functionalities may be localized into three main domains, the N-terminal, the center, and C- terminal regions; the N- and C-terminal are conserved [21, 22]. As shown in Figure 1, Atcoilin consists of three important functional domains, NOD in the N-terminal, IDD in the center, and the CTD in the C-terminal. Like many coilins, IDD of Atcoilin contains a K-rich region from 202 to 208 aa, indicating a putative nucleolar localization signal. The C-terminal of includes a Tudor-like structure. The results show that p2 of RSV binds with the full-length of Atcoilin in the nucleus, targeting to the nucleoli and Cajal bodies (Figure 3(a)). Although p2 also interacts with the IDD and CTD of Atcoilin in the nucleus, their combination failed to obviously localize in nucleolus and Cajal bodies (Figures 3(c) and 3(d)). Atcoilin localized outside the nucleus; p2 localized in the nucleus, and it unsuccessfully integrated with NOD of Atcoilin (Atcolin-1). It was reported previously that the N-terminal region of coilin was critical for CB assembly, self-interaction, and targeting to CBs and CB formation [23]. CBs can translocate outside the nucleus by separating into two daughter bodies or join to form larger bodies and maybe involve in nuclear transport events [24]. As preciously suggested, the results in the colocalization assay indicated that Atcoilin-1 form into small or big granules (CBs) and move outside the nucleus. The center fragment (IDD) of Atcoilin can target nucleoli; it is consistent with the prediction that IDD domain has a nucleolar localization signal. In BiFC assay, p2 combines with the full-length of Atcoilin localizing almost in nucleoplasm. In fact, although coilin is known as the CB signature protein, the majority of coilin is found in the nucleoplasm, not the CB [25]. p2 binds with IDD and CTD of Atcoilin in the nucleus, but failed to interact with NOD of Atcoilin.

Plant CBs have also been implicated in virus-host interactions since the mechanistic properties of CBs may be hijacked by some viruses for their own benefits. It has been shown that CB components, coilin, and fibrillarin can be used by viruses to mediate virus replication and spread [26]. Coilin (CBs) were found that it not only increased *potato virus Y* (PVY) and *turnip vein clearing virus* (TVCV) pathogenicity by facilitating replication of these viruses but also contributes to plant defense against *tobacco rattle virus* (TRV) and *tomato black ring virus* (TBRV) [1]. Some components of gene silencing machinery, such as AGO4 and Dicer-like 3, can colocalize with CBs [22, 25]. CBs may operate as processing centers in plants which generate RNA species involved in gene silencing [27]. p2 is an RNA silencing suppressor (RSS); many RSS were known as virulence factors able to intensify symptoms or promote systemic infection [28]. Our previous study indicated that p2 recruited nucleolar functions at first by interacting fibrillarin, which was a maker protein of the nucleolus, underwent necessary modification in the nucleus, and then entered to the cytoplasm to promoted RSV systemic movement [20]. Different from ORF3 of GRV, it reorganized CBs (Atcoilin) into multiple CB-like structures and then enters the nucleolus to involve in virus infection [4]. In this study, we found that if Atcoilin lack the NOD domain, p2 failed to localize into CBs, the NOD domain maybe essential for Atcoilin and p2 to target to CBs. It also implies that p2 may recruit nucleolus and move from the nucleus to the cytoplasm with the help of CBs.

Overall, the results of this study demonstrate that p2 also interacted with CBs, which are functionally associated with the nucleolus [24]. However, further studies are needed to provide our inference that p2 may manipulate nucleolar functions to obtain some benefits for its own normal function and then hijacks CBs (Atcoilin) as a vehicle to enter the cytoplasm to involve in virus infection.

## 4. Materials and Methods

### 4.1. Plant Growth Conditions

The *N. benthamiana* plants were grown and maintained in a green house at 25°C.

### 4.2. Plasmid Construction

The full-length ORF of Atcoilin, cDNA encoding three domains of Atcoilin, and RSV-p2 were amplified, respectively, by PCR using primers in Table 1, designed from *Arabidopsis thaliana coilin* and RSV sequences (GenBank accession: AY128933 and EF493228) downloaded from GenBank. The full-length and three domain fragments of Atcoilin were firstly inserted into the entry vector pDNOR221 and then destination vectors pEarleyGate101 (YFP) and pEarleyGate201-YN (YN) using Gateway recombination system [29]. pEarleyGate102-p2 (CFP-p2) and pEarleyGate201-YN (YC-p2) constructs were obtained by the same methods.

For yeast two-hybrid experiment, PCR products of RSV-p2, full-length of Atcoilin, and three domains of Atcoilin were digested with the suitable restriction enzymes individually, then ligated to the vector pGADT7 or pGBKT7 digested with the same enzymes, creating pGADT7-p2, pGBKT7-Atcoilin, pGBKT7-Atcoilin1, pGBKT7-Atcoilin2, and pGBKT7-Atcoilin3.

These constructs were confirmed by sequencing conducted by Takara (Dalian, China).

### 4.3. Yeast Two-Hybrid Assay

pGBKT7-Atcoilin, pGBKT7-Atcoilin1, pGBKT7-Atcoilin2, and pGBKT7-Atcoilin3 were introduced together with pGADT7-p2 or pGADT7. pGADT7-p2 was introduced together with pGBKT7 into the yeast strain AH109 by cotransformation. The cotransformations were selected on different SD mediums lacking tryptophan (Trp) and Leucine (Leu) (SD/Trp-Leu-); lacking histidine (His), Trp, and Leu (SD/Trp-Leu-His-); and last on the SD medium lacking adenine (Ade), His, Trp, and Leu (SD/Trp-Leu-His-Ade-).

### 4.4. Agrobacterium-Mediated Transient Expression

*A. tumefaciens* strain EHA105 were grown separately to OD_600_ = 0.8 at 28°C on Luria-Bertani liquid medium supplemented with 50 *μ*g/*μ*L of rifampicin and 50 *μ*g/*μ*L of kanamycin. The resulting cultures were centrifuged at 12,000 g for 1 min and then resuspended in induction media (10 mM MES, pH 5.6, 10 mM MgCl2, and 150 mΜ acetosyringone). In colocalization and BiFC assays, *A. tumefaciens* containing NbFib2s were separately mixed with p2 in equal volume. The mixtures of the bacterial cultures were incubated at room temperature for 3 h, then infiltrated onto fully grown upper leaves. A six-week-old *N. benthamiana* was used for the experiment.

### 4.5. Confocal Imaging Analysis

Subcellular localizations of proteins were monitored at 48 h after infiltration under a confocal microscope (Microsystems CMS GmbH Leica TCS SP5). The fluorophores in CFP and YFP were excited at 458 and 514 nm, and images were taken using BA480-495 and BA535–565 nm emission filters, respectively.

## Figures and Tables

**Figure 1:** Schematic representation of the functional domains of coilin from *Arabidopsis thaliana.* Atcoilin-1: NOD, N-terminal ordered domain from 1 aa to 117 aa; Atcoilin-2: IDD, central disordered domain from 118 aa to 350aa K-rich localizes from 202 aa to 208 aa meaning nuclear localization signals (NLS); Atcoilin-3: CTD, C-terminal domain from 351 aa to 608 aa, containing a Tudor-like structure.

**Figure 2:** Interaction analyses of p2 and Atcoilin and the three domains of Atcoilin by yeast two-hybrid (Y2H). (a) Interaction analyses between p2 and full-length of Atcoilin and (b) interaction analyses of p2 and three domains of Atcoilin. pGAD-T/pGBK-53 is a positive control. pGAD-T/pGBK-Lam is a negative control.

**Figure 3:** Subcellular colocalization of *Rice stripe virus* p2 and *Arabidopsis thaliana* coilin (Atcoilin) in epidermal cells of *Nicotiana benthamiana* at 48 h postinfiltration. (a) p2-CFP was coexpressed with Atcoilin-YFP; (b) p2-CFP was not coexpressed with Atcoilin-1-YFP; (c) p2-CFP was coexpressed with Atcoilin-2-YFP; (d) p2-CFP was coexpressed with Atcoilin-3-YFP. The nucleus was stained with 4, 6-diaminophenylindole (DAPI). Possible nucleolus or Cajal bodies described in the text are designated with red and blue arrows, respectively. Scale bars, 10 *μ*m.

**Figure 4:** Bimolecular fluorescence complementation (BiFC) assay showing interaction between p2 and Atcoilin, Atcoilin-2, and Atcoilin-3. Fluorescence was observed at 48 h postinfiltration. The nucleus was stained with 4, 6-diaminophenylindole (DAPI). Scale bars, 10 *μ*m.

**Table 1:** The sequences, homologous recombination, and restriction sites of PCR primers.

Primer and purpose	Sequence (5′→3′)^a^	Modification
Construction for yeast two-hybrid assay		
p2-ADF	CGggatccTGATGGCATTACTCCTTTTC	*Bam*HI
p2-ADR	CCGctcgagTCACATTAGAATAGGACACT	*Xho*I
Atcoilin-BDF	GgaattcATGGAGGAAGAGAAGGTGAGGTG	*EcoR*I
Atcoilin-1-BDR	CGggatccTCACCTTTCCTCAACCTCAAT	*Bam*HI
Atcoilin-2-BDF	CCcatatgATGGGCCTCAGATTCGTCCTGGTG	*Nde*I
Atcoilin-2-BDR	CGggatccTCAAGAGGCTTCATCTGTTCC	*Bam*HI
Atcoilin-3-BDF	CCcatatgATGCTTGATAGTGAACCTCTTG	*Nde*I
Atcoilin-BDR	CGggatccTCAAATCTCTTTCTGAGATC	*Bam*HI
Construction for entry vector pDONR221		
p2-GF	ggggacaagtttgtacaaaaaagcaggcttcATGGCATTACTCC TTTTC	Homologous recombination
p2-GR	ggggaccactttgtacaagaaagctgggtcCATTAGAATAGGACACT	Homologous recombination
Atcoilin-GF	ggggacaagtttgtacaaaaaagcaggcttcATGGAGGAAGAGAAGGTG	Homologous recombination
Atcoilin-1-GR	ggggaccactttgtacaagaaagctgggtcCCTTTCCTCAACCTCAAT	Homologous recombination
Atcoilin-2-GF	ggggacaagtttgtacaaaaaagcaggcttcATGGGCCTCAGATTCGTCCT	Homologous recombination
Atcoilin-2-GR	ggggaccactttgtacaagaaagctgggtcAGAGGCTTCATCTGTTCC	Homologous recombination
Atcoilin-3-GF	ggggacaagtttgtacaaaaaagcaggcttcATGCTTGATAGTGAACCTCT	Homologous recombination
Atcoilin-GR	ggggaccactttgtacaagaaagctgggtcAATCTCTTTCTGAGATC	Homologous recombination

^a^The letters in lower case indicate homologous recombination sequence or a restriction enzyme site.

## Data Availability

The full-length ORF of genes are available in GenBank. The data used to support the findings of this study are included within the article.

## References

[1] Shaw J., Love A. J., Makarova S. S., Kalinina N. O., Harrison B. D., Taliansky M. E. (2014). Coilin, the signature protein of Cajal bodies, differentially modulates the interactions of plants with viruses in widely different taxa. *Nucleus*.

[2] Boulon S., Westman B. J., Hutten S., Boisvert F. M., Lamond A. I. (2010). The nucleolus under stress. *Molecular Cell*.

[3] James N. J., Howell G. J., Walker J. H., Blair G. E. (2010). The role of Cajal bodies in the expression of late phase adenovirus proteins. *Virology*.

[4] Kim S. H., Ryabov E. V., Kalinina N. O. (2007). Cajal bodies and the nucleolus are required for a plant virus systemic infection. *The EMBO Journal*.

[5] Kim S. H., MacFarlane S., Kalinina N. O. (2007). Interaction of a plant virus-encoded protein with the major nucleolar protein fibrillarin is required for systemic virus infection. *PNAS*.

[6] Semashko M. A., Rakitina D. V., González I., Canto T., Kalinina N. O., Taliansky M. E. (2012). Movement protein of hordeivirus interacts in vitro and in vivo with coilin, a major structural protein of Cajal bodies. *Doklady. Biochemistry and Biophysics*.

[7] Cho W. K., Lian S., Kim S. M., Park S. H., Kim K. H. (2013). Current insights into research on *Rice stripe virus*. *Plant Pathology Journal*.

[8] Hibino H. (1996). Biology and epidemiology of rice viruses. *Annual Review of Phytopathology*.

[9] King A. M. Q., Adams M. J., Lefkowitz E. J., Carstens E. B. (2012). *Virus taxonomy: classification and nomenclature of virues: ninth report of the International Committee on Taxonomy of Viruses*.

[10] Falk B. W., Tsai J. H. (1998). Biology and molecular biology of viruses in the genus *Tenuivirus*. *Annual Review of Phytopathology*.

[11] Ramirez B. C., Haenni A. L. (1994). Molecular biology of tenuiviruses, a remarkable group of plant viruses. *The Journal of General Virology*.

[12] Toriyama S., Takahashi M., Sano Y., Shimizu T., Ishihama A. (1994). Nucleotide sequence of RNA 1, the largest genomic segment of rice stripe virus, the prototype of the *tenuiviruses*. *The Journal of General Virology*.

[13] Kong L., Wu J., Lu L., Xu Y., Zhou X. (2014). Interaction between Rice stripe virus disease-specific protein and host PsbP enhances virus symptoms. *Molecular Plant*.

[14] Xu Y., Zhou X. (2012). Role of rice stripe virus NSvc4 in cell-to-cell movement and symptom development in *Nicotiana benthamiana*. *Frontiers in Plant Science*.

[15] Zhang C., Pei X., Wang Z. (2012). The Rice stripe virus pc4 functions in movement and foliar necrosis expression in *Nicotiana benthamiana*. *Virology*.

[16] Xiong R., Wu J., Zhou Y., Zhou X. (2009). Characterization and subcellular localization of an RNA silencing suppressor encoded by *Rice stripe tenuivirus*. *Virology*.

[17] Hayakawa T., Zhu Y., Itoh K. (1992). Genetically engineered rice resistant to rice stripe virus, an insect-transmitted virus. *PNAS*.

[18] Zhao S. L., Dai X. J., Liang J. S., Liang C. Y. (2012). Surface display of rice stripe virus NSvc2 and analysis of its membrane fusion activity. *Virologica Sinica*.

[19] Du Z., Xiao D., Wu J. (2011). p2 of *Rice stripe virus* (RSV) interacts with OsSGS3 and is a silencing suppressor. *Molecular Plant Pathology*.

[20] Zheng L., Du Z., Lin C. (2015). Rice stripe tenuivirus p2 may recruit or manipulate nucleolar functions through an interaction with fibrillarin to promote virus systemic movement. *Molecular Plant Pathology*.

[21] Tucker K. E., Massello L. K., Gao L. (2000). Structure and Characterization of the Murine p80 Coilin Gene, *Coil*. *Journal of Structural Biology*.

[22] Makarov V., Rakitina D., Protopopova A. (2013). Plant coilin: structural characteristics and RNA-binding properties. *PLoS One*.

[23] Hebert M. D., Matera A. G. (2000). Self-association of coilin reveals a common theme in nuclear body localization. *Molecular Biology of the Cell*.

[24] Ogg S. C., Lamond A. I. (2002). Cajal bodies and coilin—moving towards function. *The Journal of Cell Biology*.

[25] Lam Y. W., Lyon C. E., Lamond A. I. (2002). Large-scale isolation of Cajal bodies from HeLa cells. *Molecular Biology of the Cell*.

[26] Love A. J., Yu C., Petukhova N. V., Kalinina N. O., Chen J., Taliansky M. E. (2017). Cajal bodies and their role in plant stress and disease responses. *RNA Biology*.

[27] Bassett C. L. (2012). Cajal bodies and plant RNA metabolism. *Critical Reviews in Plant Sciences*.

[28] Díaz-Pendón J. A., Ding S. W. (2008). Direct and indirect roles of viral suppressors of RNA silencing in pathogenesis. *Annual Review of Phytopathology*.

[29] Karimi M., Inzé D., Depicker A. (2002). GATEWAY™ vectors for *Agrobacterium*-mediated plant transformation. *Trends in Plant Science*.

